RETRACTED

# Downregulation of OIP5-AS1 affects proNGF-induced pancreatic cancer metastasis by inhibiting p75NTR levels

**DOI:** 10.18632/aging.202847

**Published:** 2021-04-03

**Authors:** Ang Li, Lei Feng, Xiaoya Niu, Qihui Zeng, Bei Li, Zhen You

**Affiliations:** 1 Department of Pancreatic Surgery, West China Hospital of Sichuan University, Chengdu 610041, China; 2 Department of Biliary Surgery, West China Hospital of Sichuan University, Chengdu 610041, China

**Keywords:** pancreatic cancer, long non-coding RNA OIP5-AS1, microRNA-186-5p, nerve growth factor receptor, pro-nerve growth factor

## Abstract

We aimed to explore the mechanism by which long non-coding RNA (lncRNA) OIP5-AS1 affects proNGF (precursor nerve growth factor)-induced pancreatic cancer metastasis by targeting the miR-186-5p/NGFR axis. Bioinformatics was used to analyse whether OIP5-AS1 targets miR-186-5p/NGFR and their expression characteristics in pancreatic cancer. OIP5-AS1 and NGFR were overexpressed in pancreatic cancer, and their levels showed a significant positive correlation. Clinical trials also demonstrated that high expression of OIP5-AS1 and NGFR and low expression of miR-186-5p played a pro-cancer role in pancreatic cancer. MiR-186-5p inhibited the migration and invasion of colon cancer cells by targeting NGFR-regulated p75NTR. OIP5-AS1 regulated the action of miR-186-5p on NGFR mRNA and p75NTR by targeting miR-186-5p. Downregulation of NGFR inhibited the expression of p75NTR protein and blocked the role of proNGF in promoting the migration and invasion of pancreatic cancer cells. Animal experiments also showed that the knockdown of miR-186-5p promoted cancer via the expression of NGFR mRNA and p75NTR protein, while the downregulation of proNGF blocked the effects. OIP5-AS1, as a ceRNA, promotes the progression of pancreatic cancer by targeting miR-186-5p/NGFR and affecting the prognosis of patients, which may be related to the action of proNGF.

## INTRODUCTION

As a more common clinical digestive tract tumour, pancreatic cancer has the characteristics of high malignancy and a poor prognosis [1]. The incidence of pancreatic cancer is high, and the survival rate of patients is not ideal [2]. Because the early symptoms of pancreatic cancer are not obvious, most patients are already in an advanced stage at the time of diagnosis, missing the best chance of surgery [3, 4]. The high metastatic potential of pancreatic cancer is an important factor affecting the poor prognosis of pancreatic cancer [5–7]. Therefore, the analysis of the molecular mechanism of pancreatic cancer metastasis is the basis for developing new treatment methods.

Long non-coding RNAs (lncRNAs) comprise more than 200 nucleotides in length and do not have protein translation capabilities [8, 9]. LncRNAs can target microRNAs (miRNAs) as competing endogenous RNAs (ceRNAs), thereby regulating the role of miRNAs in the degradation and translation of messenger RNA (mRNA) [10–12]. Studies have found that lncRNAs play an important role in tumour apoptosis, metastasis, and drug resistance [13–15]. OIP5-AS1 is a newly discovered lncRNA closely related to tumours that regulates the expression of target genes by targeting miRNAs and the occurrence and development of multiple myeloma, colorectal cancer, and lung adenocarcinoma, among other cancers [16–18]. However, the role of OIP5-AS1 in pancreatic cancer remains unclear.

RETRACTED

Nerve growth factor (NGF) is an active substance that is cleaved from its precursor proNGF and is involved in the growth, differentiation and development of neurons [19, 20]. ProNGF was initially considered to be inactive, but recent research has found that proNGF has biological activity independent of NGF [21–23]. proNGF is involved in the development and progression of tumours by binding to its receptors tyrosine kinase A (TrkA) and p75 neurotrophin receptor (p75NTR) [24–26]. Downregulation of the proNGF levels inhibits the proliferation and invasion of pancreatic cancer cells [27]. ProNGF promotes the invasiveness of breast cancer cells by binding to TrkA receptors [24]. NGFR encodes the p75NTR protein, and overexpression of p75NTR promotes the invasion of pancreatic cancer cells to peripheral nerves [28]. A recent study showed that p75NTR is significantly upregulated in patients with oesophageal cancer as a tumour marker [29]. Overexpression of NGFR increases the invasion and metastasis of oral squamous cell carcinoma [30].

In this study, we found that OIP5-AS1 is associated with a poor prognosis of pancreatic cancer cells and is significantly positively correlated with the NGFR levels by bioinformatics analysis. Furthermore, the mechanisms by which OIP5-AS1 regulates pancreatic cancer cell metastasis by targeting the miR-186-5p/NGFR axis and affects proNGF in pancreatic cancer cells by regulating NGFR expression were further analysed.

## RESULTS

### OIP5-AS1 is associated with a poor prognosis of pancreatic cancer and is positively associated with NGFR

Initially, by bioinformatics analysis, we found that OIP5-AS1 was overexpressed in patients with pancreatic cancer and was associated with a poor prognosis (Figure 1A, 1B). Furthermore, NGFR was also overexpressed in pancreatic cancer, and co-expression analysis showed that the levels of OIP5-AS1 and NGFR showed a significant positive correlation in pancreatic cancer (Figure 1C–1E).

**Figure 1:** **OIP5-AS1 is associated with a poor prognosis of pancreatic cancer and is positively associated with NGFR.** (**A**) Expression characteristics of OIP5-AS1 in pancreatic cancer. (**B**) Relationship between OIP5-AS1 and the survival rate. (**C**) Expression characteristics of NGFR in pancreatic cancer. (**D**, **E**) Relationship between OIP5-AS1 and NGFR.

RETRACTED

### OIP5-AS1 is involved in the regulation of NGFR by miR-186-5p

Bioinformatics analysis also showed that miR-186-5p was under-expressed in pancreatic cancer and negatively correlated with OIP5-AS1 (Figure 2A, 2B). Moreover, we found that low miR-186-5p levels were associated with a poor prognosis in pancreatic cancer (Figure 2C). Next, we performed differential analysis of GSE28735 and obtained 250 upregulated genes. The potential target genes of miR-186-5p were predicted, and 97 genes were obtained by overlapping with the upregulated genes (Figure 2D). Gene Ontology (GO) analysis of these 97 genes revealed that NGFR was enriched in the integral component of plasma membrane and is the main component of the cell membrane. Additionally, miR-186-5p-related target genes were mainly enriched in pathways associated with the extracellular matrix and cell adhesion (Figure 2E, 2F).

**Figure 2:** **OIP5-AS1 is involved in the regulation of NGFR by miR-186-5p.** (**A**) Expression characteristics of miR-186-5p in pancreatic cancer. (**B**) Relationship between OIP5-AS1 and miR-186-5p. (**C**) Relationship between miR-186-5p and the survival rate. (**D**) Venn diagram of the upregulated genes in GSE28735 and target gene of miR-186-5p. (**E**, **F**) GO analysis of 97 common genes.

### OIP5-AS1 directly targets miR-186-5p, and miR-186-5p directly targets NGFR

The website (http://starbase.sysu.edu.cn/index.php) predicted the binding site of OIP5-AS1 targeting miR-186-5p and miR-186-5p targeting NGFR (Figure 3A, 3B). The level of miR-186-5p was significantly increased after the transfection of miR-186-5p mimic (Figure 3C). Dual luciferase reporter assay results confirmed that OIP5-AS1 directly targeted miR-186-5p, and miR-186-5p directly targeted NGFR (Figure 3D, 3E). Thus, miR-186-5p targets NGFR, while OIP5-AS1 regulates NGFR and p75NTR by targeting miR-186-5p.

**Figure 3:** **OIP5-AS1 directly targets miR-186-5p, and miR-186-5p directly targets NGFR.** (**A**, **B**) Targeted binding site of OIP5-AS1/miR-186-5p and miR-186-5p/NGFR. (**C**) Level of miR-186-5p after transfection. (**D**, **E**) Results of the dual luciferase reporter assay. ^*^P < 0.05 vs. mimic-NC group.

### OIP5-AS1, NGFR and miR-186-5p are associated with the prognosis in patients with pancreatic cancer

Analysis of clinical samples of pancreatic cancer showed that OIP5-AS1 was significantly upregulated and miR-186-5p was significantly downregulated (Figure 4A, 4B). Additionally, the expression levels of NGFR mRNA and protein in pancreatic cancer tissues were also significantly higher than those in adjacent tissues (Figure 4C, 4D). Moreover, immunohistochemical staining results showed that the level of p75NTR protein encoded by NGFR in pancreatic cancer tissues was significantly higher than that in normal tissues (Figure 4E). In pancreatic cancer tissues, the level of miR-186-5p was negatively correlated with the levels of OIP5-AS1 and NGFR, respectively, and OIP5-AS1 and NGFR were positively correlated (Figure 4F–4H). Furthermore, survival analysis showed that pancreatic cancer patients with high expression of OIP5-AS1 and NGFR had low survival rates, while patients with low expression of miR-186-5p had a lower survival rate (Figure 4I–4K). Clinical trials also demonstrated that high expression of OIP5-AS1 and NGFR and low expression of miR-186-5p played a pro-cancer role in pancreatic cancer.

RETRACTED

**Figure 4:** **OIP5-AS1, NGFR and miR-186-5p are associated with prognosis in patients with pancreatic cancer.** (**A**–**D**) Expression characteristics of OIP5-AS1, miR-186-5p and NGFR in pancreatic cancer patients. (**E**) Levels of p75NTR protein encoded by NGFR in pancreatic cancer and normal tissues (×100). (**F**–**H**) Correlation between the OIP5-AS1, miR-186-5p and NGFR levels. (**I**–**K**) Relationship between the OIP5-AS1, miR-186-5p and NGFR levels and survival rate in patients with pancreatic cancer.

### MiR-186-5p inhibits the migration and invasion of pancreatic cancer by targeting NGFR.

First, we verified the establishment of NGFR-overexpressing cell lines by qPCR and Western blotting (Figure 5A, 5B). To analyse the effects of miR-186-5p targeting NGFR on pancreatic cancer cells, Panc-1 and Capan-1 cells were divided into 4 groups: si-NC + inhibitor-NC, si-NC + inhibitor-miR-186-5p, si-NGFR + inhibitor-miR-186-5p and si-NGFR + inhibitor-NC. Downregulation of the miR-186-5p levels promoted cell viability in Panc-1 and Capan-1 cells. Knocking down NGFR inhibited cell viability and partially reversed the promotion of cell viability by low miR-186-5p expression (Figure 5C, 5D). In Panc-1 cells, knocking down miR-186-5p increased the ability of cells to migrate and invade. Downregulation of NGFR resulted in the decreased migration and invasion ability of Panc-1 cells and partially reversed the promotion of low miR-186-5p expression on migration and invasion (Figure 5E, 5F). The effects of miR-186-5p and NGFR on Capan-1 cells had the same trend as those on Panc-1 cells (Figure 5G, 5H), indicating that miR-186-5p inhibited the migration and invasion of colon cancer cells by targeting NGFR-regulated p75NTR.

RETRACTED

**Figure 5:** **MiR-186-5p inhibits the migration and invasion of pancreatic cancer by targeting NGFR.** (**A**, **B**) Levels of NGFR mRNA and p75NTR protein after transfection. (**C**, **D**) Comparison of the cell viability in each group. (**E**, **F**) Comparison of the migration and invasion abilities of Panc-1 cells in different groups. (**G**, **H**) Comparison of the migration and invasion abilities of Capan-1 cells in different groups.

### OIP5-AS1 promotes migration and invasion by targeting the miR-186-5p/NGFR axis

We verified the establishment of OIP5-AS1 overexpressing cell lines by qPCR (Figure 6A, 6B). Panc-1 and Capan-1 cells were divided into 4 groups: si-NC + inhibitor-NC, si-OIP5-AS1 + inhibitor-NC, si-OIP5-AS1 + inhibitor-miR-186-5p and si-NC + inhibitor-miR-186-5p. Downregulation of the OIP5-AS1 levels inhibited cell viability in Panc-1 and Capan-1 cells. Knocking down miR-186-5p promoted cell viability and partially reversed the inhibition of cell viability by OIP5-AS1 low expression (Figure 6C, 6D). In Panc-1 cells, knocking down OIP5-AS1 decreased the ability of cells to migrate and invade. Downregulation of miR-186-5p resulted in the increased migration and invasion ability of Panc-1 cells and partially reversed the inhibition effects of low miR-186-5p expression on migration and invasion (Figure 6E, 6F). The effects of OIP5-AS1 and miR-186-5p on Capan-1 cells showed the same trend as those on Panc-1 cells (Figure 6G, 6H). Additionally, the results showed that the downregulation of OIP5-AS1 levels inhibited NGFR mRNA and p75NTR expression and the knockdown miR-186-5p partially reversed the inhibitory effects of low OIP5-AS1 expression on NGFR and p75NTR expression (Figure 6I–6L). These findings suggest that OIP5-AS1 regulates the action of miR-186-5p on NGFR mRNA and p75NTR by targeting miR-186-5p, thereby participating in the migration and invasion of pancreatic cancer.

**Figure 6:** **OIP5-AS1 promotes migration and invasion by targeting the miR-186-5p/NGFR axis.** (**A**, **B**) Level of OIP5-AS1 and miR-186-5p protein after transfection. (**C**, **D**) Comparison of cell viability in each group. (**E**, **F**) Comparison of the migration and invasion abilities of Panc-1 cells in different groups. (**G**, **H**) Comparison of the migration and invasion abilities of Capan-1 cells in different groups. (**I**–**L**) Comparison of the NGFR mRNA and p75NTR protein levels in each group.

### P75NTR plays a role in promoting cancer by combining with proNGF

First, we confirmed the successful establishment of Panc-1 and Capan-1 cells with overexpression of proNGF by Western blotting (Figure 7A). To analyse the role of p75NTR in proNGF-promoting pancreatic cancer cell migration and invasion, Panc-1 and Capan-1 cells were divided into 3 groups: OE-NC + si-NC, OE-proNGF + si-NC and OE-proNGF + si-NGFR. The up-regulation of proNGF levels promoted cell viability, while knocking down NGFR to reduce p75NTR protein expression partially reversed the promotion of proNGF in colon cancer cells. After knocking down NGFR, the cell viability was reduced to a level comparable to that of the control group (Figure 7B, 7C). In Panc-1 cells, overexpression of proNGF increased the ability of cells to migrate and invade, while knocking down NGFR partially reversed the promotion of migration and invasion by proNGF (Figure 7D, 7E). This trend was also shown in Capan-1 cells (Figure 7F, 7G). Thus, the downregulation of NGFR inhibits the expression of p75NTR protein and blocks the role of proNGF in promoting the migration and invasion of pancreatic cancer cells.

RETRACTED

**Figure 7:** **P75NTR plays a role in promoting cancer by combining with proNGF.** (**A**) Level of proNGF after transfection. (**B**, **C**) Comparison of the cell viability in each group. (**D**, **E**) Comparison of the migration and invasion abilities of Panc-1 cells in different groups. (**F**, **G**) Comparison of the migration and invasion abilities of Capan-1 cells in different groups.

### OIP5-AS1 regulates the role of proNGF in promoting cell migration and invasion by targeting the miR-186-5p/NGFR axis

To demonstrate the mechanism by which OIP5-AS1 regulates NGFR expression by targeting miR-186-5p, Panc-1 cells were divided into three groups, si-NC + inhibitor-NC, si-OIP5-AS1 + inhibitor-NC and si-OIP5-AS1 + inhibitor-miR-186-5p. The transfected cells were used to carry out a tumour-bearing nude mouse model. The results showed that OIP5-AS1 knockdown significantly inhibited tumour growth, while knocking down miR-186-5p partially reversed the inhibitory effects of low OIP5-AS1 expression on tumour growth (Figure 8A). The levels of OIP5-AS1 and NGFR mRNA in tumour tissues in the si-OIP5-AS1 + inhibitor-NC group were significantly lower than those in the si-NC + inhibitor-NC group, and the level of miR-186-5p was significantly higher than that in the si-NC + inhibitor-NC group. The OIP5-AS1 and NGFR mRNA levels in the si-OIP5-AS1 + inhibitor-miR-186-5p group were significantly higher than those in the si-OIP5-AS1 + inhibitor-NC group, and the miR-186-5p level was significantly lower than that in the si-OIP5-AS1 + inhibitor-NC group (Figure 8B). Additionally, the level of p75NTR protein in the three groups was the same as the NGFR mRNA level (Figure 8C). Thus, OIP5-AS1 regulates the expression of NGFR mRNA and p75NTR protein by targeting miR-186-5p.

RETRACTED

**Figure 8:** **OIP5-AS1 regulates the role of proNGF in promoting cell migration and invasion by targeting the miR-186-5p/NGFR axis.** (**A**) Comparison of the tumour weight of mice in each group. (**B**, **C**) OIP5-AS1, miR-186-5p, NGFR mRNA and p75NTR protein levels of tumour tissues in each group. (**D**) Comparison of the tumour weight of mice in each group. (**E**, **F**) Levels of miR-186-5p, NGFR and proNGF mRNA, and p75NTR and proNGF proteins in the tumour tissues of each group.

Capan-1 cells were divided into 4 groups: inhibitor-NC + si-NC, inhibitor-miR-186-5p + si-NC, inhibitor-miR-186-5p + si-proNGF and inhibitor-NC + si-proNGF. The tumour-bearing nude mice model was constructed by subcutaneous injection, with 4 mice in each group. The results showed that the knockdown of miR-186-5p promoted tumour growth while knocking down proNGF inhibited tumour growth. Additionally, knocking down proNGF partially reversed the effects of miR-186-5p low expression on tumour growth (Figure 8D). The miR-186-5p of the inhibitor-miR-186-5p + si-NC group was slightly decreased while the NGFR mRNA and p75NTR protein were significantly increased. Additionally, the level of proNGF mRNA was not significantly changed. Thus, miR-186-5p was targeted to inhibit NGFR and had no significant effect on proNGF (Figure 8E, 8F). These findings showed that the knockdown of miR-186-5p promoted cancer by promoting the expression of NGFR mRNA and p75NTR protein, while the downregulation of proNGF blocked the effects. Thus, the downregulation of NGFR mRNA and p75NTR protein expression might affect the promotion of pancreatic cancer by proNGF.

## DISCUSSION

In this study, we found that OIP5-AS1 regulated the expression of NGFR mRNA and p75NTR protein by targeting miR-186-5p and regulated the migration and invasion of pancreatic cancer cells. The downregulation of NGFR mRNA and p75NTR protein might affect the role of proNGF in promoting pancreatic cancer progression.

The role of lncRNAs in pancreatic cancer has been discovered. For example, NUTF2P3-001, UCA1, and GAS5 participate in the occurrence, development, metastasis and drug resistance by ceRNA [31–33]. OIP5-AS1 acts as a biomarker for bladder cancer and oral tumours [34, 35]. In lung cancer, hepatoblastoma, melanoma, and osteosarcoma, OIP5-AS1 acts as a ceRNA and regulates miRNA and target genes to promote proliferation, metastasis and drug resistance [36–39]. However, the role of OIP5-AS1 in pancreatic cancer remains elusive. In this study, we found that OIP5-AS1 was overexpressed in patients with pancreatic cancer by bioinformatics analysis. Patients with high levels of OIP5-AS1 had a poor prognosis, and OIP5-AS1 was positively correlated with the NGFR levels. Thus, OIP5-AS1 may be involved in the progression of pancreatic cancer. Moreover, OIP5-AS1 directly targets miR-186-5p and subsequent clinical trials have confirmed that OIP5-AS1 was upregulated and miR-186-5p was downregulated in patients with pancreatic cancer. OIP5-AS1 and miR-186-5p showed a negative correlation: high OIP5-AS1 levels and low miR-186-5p levels were associated with a poor prognosis. Furthermore, OIP5-AS1 directly targeted miR-186-5p. To further analyse the role of OIP5-AS1 and miR-186-5p in the progression of pancreatic cancer, we performed differential analysis of GSE28735. The obtained upregulated genes were co-assembled with the potential target gene of miR-186-5p to obtain 97 common genes. These genes were found to be primarily involved in extracellular matrix or migration and invasion by GO analysis. Therefore, we conclude that OIP5-AS1 may be involved in the migration and invasion of pancreatic cancer by regulating the miR-186-5p/NGFR axis.

RETRACTED

MiR-186-5p is a miRNA whose role in tumours is gradually emerging. MiR-186-5p plays a tumour suppressor role in osteosarcoma, colorectal cancer and cholangiocarcinoma [40–42]. Moreover, the process by which miR-186-5p targets genes is regulated by lncRNA [43, 44]. In this study, we verified that miR-186-5p inhibited the migration and invasion of colon cancer cells by inhibiting the level of NGFR. OIP5-AS1 negatively regulated miR-186-5p-targeted NGFR and the effects on cells by targeting miR-186-5p. Thus, in pancreatic cancer, OIP5-AS1 promotes the migration and invasion of pancreatic cancer by targeting miR-186-5p/NGFR.

The p75NTR protein is encoded by NGFR. Previous studies have shown that p75 (NGFR) is involved in the invasion of pancreatic cancer to peripheral nerves [28]. Bapat’s findings [45] also showed that decreasing p75NTR expression inhibits pancreatic cancer cell- nerve invasion. Additionally, p75NTR may be the starting gene for tetraglioma [46]. However, the p75NTR-proNGF pathway may promote apoptosis by inducing natural killer cells [47]. Kojima [48] showed that p75NTR inhibited the mitosis of oesophageal squamous cell carcinoma cells and increased stem cell characteristics. Our study showed that the upregulation of proNGF levels promoted the ability of pancreatic cancer cells to migrate and invade, while the downregulation of the p75NTR protein levels blocked the pro-cancer effects of proNGF. Thus, p75NTR promotes migration and invasion by binding to its ligand proNGF.

Subsequent animal experiments also showed that OIP5-AS1 promotes the expression of NGFR mRNA and p75NTR protein by targeting miR-186-5p and promoting tumour growth in tumour-bearing nude mice. Additionally, the downregulation of miR-186-5p promotes tumour growth by promoting the expression of NGFR mRNA and p75NTR protein, whereas proNGF partially reverses the effect of miR-186-5p/NGFR on tumour growth. Thus, OIP5-AS1 regulates the expression of NGFR mRNA and p75NTR protein by targeting miR-186-5p, thereby affecting the effect of proNGF on cells. This effect is a complex process; proNGF can be cleaved to generate NGF, and NGF can also play a biological role by combining with TrkA and p75NTR [49, 50]. Minnone [51] showed that proNGF, rather than NGFR, promoted chronic inflammation through p75NTR rather than TrkA. proNGF is generally combined with p75NTR instead of TrkA, but proNGF can promote apoptosis in response to decreased levels of TrkA [52]. Our study demonstrated that OIP5-AS1 might affect the migration and invasion of pancreatic cancer cells by regulating miR-186-5p/NGFR. However, further studies are needed to elucidate the relationship between the proNGF/p75NTR pathway and NGF and TrkA, and their mechanisms in regulating migration and invasion.

RETRACTED

In summary, OIP5-AS1, as a ceRNA, could promote the progression of pancreatic cancer by targeting miR-186-5p/NGFR and affecting the prognosis of patients, findings that might be related to the action of proNGF. However, further study is needed on the mechanism by which OIP5-AS1, particularly NGFR, is involved in pancreatic cancer metastasis.

## MATERIALS AND METHODS

### Bioinformatics analysis

The expression characteristics of OIP5-AS1, miR-186-5p and NGFR in pancreatic cancer patients in The Cancer Genome Atlas (TCGA) database were analysed using the website tools GEPIA (http://gepia.cancer-pku.cn/index.html) and Starbase (http://starbase.sysu.edu.cn/index.php). GSE28735 in the GEO database was downloaded. GSE28735 compares the genomes of pancreatic patients with different prognoses. Limma was used for differential analysis, and the differential expression conditions were set as follows: log|FC| > 1 and P <0.05. The predicted results of the target genes were from Starbase.

### Clinical research

The cancer and normal tissue samples of 86 pancreatic cancer patients were collected. All the patients did not receive radiotherapy or chemotherapy within 3 months before enrolment. The levels of OIP5-AS1, miR-186-5p and NGFR in the tissue were detected by quantitative polymerase chain reaction (qPCR) and/or Western blotting.

### Cell culture and transfection

The pancreatic cancer cell lines Panc-1 and Capan-1 (American Type Culture Collection, USA) were cultured in RPMI-1640 medium containing 10% foetal bovine serum (FBS; Thermo Fisher, Waltham, MA, USA), 50 U/mL of penicillin and 50 μg/mL of streptomycin (15070063; Thermo Fisher, Waltham, MA, USA). Plasmid transfection was used to knock down or overexpress genes. Briefly, 2 μL of Lipofectamine^TM^ 2000 (Invitrogen, Waltham, USA) and 40 pmol of plasmid or negative control (NC) (GenePharma) were mixed in 50 μL of serum-free medium at room temperature for 15 min. The lipid compounds were diluted in 300 μL of serum-free medium and 600 μL of medium containing FBS to produce a 1-mL volume mixture, which was incubated with the cells at 37° C in 5 % CO_2_ for subsequent experiments.

RETRACTED

### Qpcr

Total RNAs were isolated using TRIzol reagent (Invitrogen, Waltham, USA). The concentration and purity of the RNA were examined using a NanoDrop2000 spectrophotometer (Nano Drop Technologies, Wilmington, DE, USA). The RNA was reverse transcribed using a reverse transcription cDNA kit (Thermo Fisher Scientific, Waltham, USA) for cDNA synthesis (42° C for 60 min, 70° C for 5 min and then 4° C preservation). The SYBR Green PCR Master Mix (Roche, Basle, Switzerland) and PCR Detection System (ABI 7500; Life Technologies, USA) were applied to conduct qPCR. The PCR cycle parameters were as follows: pretreatment at 95° C for 10 min, followed by 40 cycles of 94° C for 15 s, 60° C for 1 min, a final incubation at 60° C for 1 min and then at 4° C for preservation. Comparative cycle threshold (ΔΔCt) was employed to analyse the RNA expression. GAPDH and U6 expression levels were used for normalisation. The primers were designed and synthesised by Genecopoeia (Guangzhou, China).

### Dual luciferase reporter assay

Wild-type OIP5-AS1 and NGFR and mutated (mut) OIP5-AS1 and NGFR constructs were cloned into pMIR-REPORT Luciferase vectors (Ambion; Thermo Fisher Scientific, Waltham, MA, USA). HEK293T cells were seeded in 6-well plates and then transfected with both vectors using Lipofectamine 2000 for 24 h. The Dual Luciferase-Reporter 1000 Assay System (Promega, Madison, WI, USA) was used to evaluate luciferase activity.

### Immunohistochemical staining

Immunohistochemical staining was applied to detect the expression of p75NTR in cancer and normal tissues. The samples were dehydrated, transparentised, immersed in wax with a gradient alcohol series and embedded in paraffin. After freezing for 20 min, the samples were cut into 4-μm sections. Next, the sections were routinely deparaffinised, hydrated and subjected to antigen retrieval, and 3% hydrogen peroxide solution (hydrogen peroxide: pure water = 1:9) was added to block endogenous peroxidase. Next, 3% BSA was added to evenly cover the tissue, which was blocked for 30 min at room temperature. A 1:100 dilution of the p75NTR antibody (ab52987; 45 kD; Abcam, San Francisco, CA, USA) was added and incubated at 37° C for 60 min. After washing, 100 μL of enhanced enzyme-labelled goat anti-rabbit IgG polymer was added to cover the tissue, which was incubated at room temperature for 60 min. DAB was applied for colour development for 5–6 min, and then the tissue was stained with haematoxylin for 20 min, dehydrated and mounted. The staining results were observed using a microscope (×100).

RETRACTED

### Cell counting kit 8 (CCK-8) assay

The cells were adjusted to a density of 2 × 10^4^ cells/mL and inoculated into 96-well plates (100 μL per well). At 48 h after transfection, 10 μL of CCK-8 (Beyotime Institute of Biotechnology, Beijing, China) was added and cultured at 37° C for 2 h. The optical density (OD) at 450 nm was measured using a microplate reader (Tecan Infinite M200 Micro Plate Reader; LabX, Männedorf, Switzerland) to calculate the relative cell viability.

### Wound healing assay

The cells were gathered and seeded in a 6-well plate (1 ×10^6^ per well) and cultured until 90% confluence in each well with medium. The cell monolayers were vertically scratched using the tip of a 200-μL pipette. The monolayers were then washed to remove cellular debris and further cultured for an additional 24 h. The monolayer images were captured under an inverted microscope (Olympus IX71; Tokyo, Japan) following wounding.

### Transwell assay

In total, 3 × 10^4^ cells were transferred to the upper chamber of a Transwell apparatus (8-μm; BD Biosciences, CA, USA). As a chemoattractant, the bottom chamber was filled with complete medium supplemented with 10% FBS. After 48 h of incubation, the cells that did not invade through the membrane were collected. The cells were then fixed with 20% methanol and stained with 0.2% crystal violet. Cells invaded into the bottom chamber per field were counted under an inverted microscope.

### Western blotting

The proteins were extracted using RIPA lysis buffer, and the BCA kit was used to analyse the protein concentration. Proteins were separated by SDS-PAGE at 110 V for 100 min and then transferred to a PVDF membrane at 90 V for 90 min. The PVDF membrane was blocked in 5% non-fat milk for 1 h at room temperature. The antibodies (p75NTR: ab52987, 45 kD, Abcam, San Francisco, CA, USA; proNGF: ALO-ANT-005-25, Alomone Inc., Israel) were diluted at 1:1000 with 5% BSA and added to the cells overnight at 4° C. Next, the secondary antibodies (sc-516102/sc-2357; Santa Cruz Biotechnology, Inc., Dallas, TX, USA) were diluted at 1:5000 and added to the cells at room temperature for 2 h. Protein bands were detected using the Pierce™ ECL plus Western blotting substrate (Thermo Fisher, Waltham, MA, USA) in ChemiDoc MP (Bio-Rad, CA, USA).

RETRACTED

### Tumour burden assay

The animal experiment protocol was approved by the Animal Experimentation Ethics Committee of West China Hospital of Sichuan University. Specific pathogen-free (SPF) 4-week-old BALB/c nude mice were purchased from the Animal Center of Air Force Medical University (Shanghai, China). The cultured cells obtained after transfection were used to generate the model. The mice were injected with 1×10^6^ cells as indicated. Twenty-eight days after injection, the mice were sacrificed, and the tumours were removed to weigh and take photos.

### Statistical analysis

All the experimental data were presented as means ± SD, and P < 0.05 was considered statistically significant. All the statistical analyses were performed using GraphPad Prism 7.

### Ethics approval and consent to participate

Following the approval of the ethical committee of West China Hospital of Sichuan University and the Helsinki Declaration, the cancer and normal tissue samples of 86 pancreatic cancer patients were collected. All the patients did not receive radiotherapy or chemotherapy within 3 months before enrolment. Written informed consent was obtained from all the participants before the study. The animal studies were performed according to the National Institutes of Health’s Guidelines for the Care and Use of Laboratory Animals and were granted approval by the Animal Care and Research Committee of West China Hospital of Sichuan University.
